# Maximizing energy storage in Microgrids with an amended multi-verse optimizer

This article has been retracted.

**DOI:** 10.1016/j.heliyon.2023.e21471

**Published:** 2023-10-24

**Authors:** Qingpu Hu, Guoxin Zhao, Jian Hu, Navid Razmjooy

**Affiliations:** a Department of Electrical Engineering, Yellow River Conservancy Technical Institute, Kaifeng, Henan, 475004, China; b Young Researchers and Elite Club, Ardabil Branch, Islamic Azad University, Ardabil, Iran; c Department of Computer Science and Engineering, Division of Research and Innovation, Saveetha School of Engineering, SIMATS, Chennai, 602105, Tamil Nadu, India; d College of Technical Engineering, The Islamic University, Najaf, Iraq

**Keywords:** Combined cooling heating and power (CCHP), Microgrid, Energy storage, Amended multi-verse optimizer algorithm (AMVOA)

## Abstract

Microgrids have emerged as a possible alternative to overcome the difficulties of the combined cooling, heating, and power (CCHP) system in power networks. Energy storage devices are vital for the stable and effective functioning of Microgrids. In this paper, a new modified metaheuristic technique, called the Amended Multiverse Optimizer algorithm (AMVOA) is used to suggest a new method of Microgrid design with energy storage. The Multiverse theory notion served as the inspiration for the metaheuristic optimization method known as the AMVOA. The suggested strategy takes into account the load demand, energy storage technologies, and architecture of a Microgrid with renewable energy sources. The goal is to keep the Microgrid's overall cost as low as possible while preserving its dependability and sustainability. To validate the efficiency of the proposed method, two HRES scenarios are put out, the first of which relies on PV, wind, diesel, and battery power, and the second of which uses PV, diesel, and battery power. To validate the superiority of the proposed method, the method has been compared with five state-of-the-art algorithms, including the Evolutionary Algorithm (EA), Modified Grasshopper Optimization Algorithm (MGOA), Improved Gray Wolf Optimization Algorithm (IGWOA), Improved Arithmetic Optimization Algorithm (IAOA), and the original MVOA. The study compares two scenarios: one with wind, PV, diesel, and battery power and the other with only PV, diesel, and battery power. In scenario 1 (Wind/PV/DG/BESS), the AMVOA algorithm achieves optimal results, resulting in a Net Present Cost (NPC) of $299,010 and an energy cost of $0.2309 per kilowatt-hour. The proposed technique successfully integrates 84.86 % renewable energy sources while meeting defined limitations. The optimal sizing for scenario 2 (PV/DG/BESS) is $333,800 with an energy cost of $0.3451 per kilowatt-hour. The AMVOA algorithm outperforms other algorithms in convergence and provides efficient power management. However, further analysis and evaluation are necessary to assess the robustness, practicality, and reliability of the proposed Microgrid configurations. The outcomes show how the suggested AMVO-based strategy may be used to create the best Microgrid architecture with energy storage. The recommended method may be applied as a decision-making tool for Microgrid planning and design, especially for the integration of renewable energy.

## List of abbreviations

**Abbreviation**
CCHP: Combined Cooling Heating and Power
AMVOA: Amended Multi-Verse Optimizer Algorithm
EA: Evolutionary Algorithm
MGOA: Modified Grasshopper Optimization Algorithm
IGWOA: Improved Gray Wolf Optimization Algorithm
IAOA: Improved Arithmetic Optimization Algorithm
LP: Linear Programming
AOA: Arithmetic Optimization Algorithm
AO: The Aquila Optimizer
EO: Equilibrium Optimizer
GWO: Gray Wolf Optimization
AEFA: Artificial Electric Field Algorithm
HHO: Harris Hawks Optimization
LCOE: Levelized Cost of Electricity
PC: Present Cost
PB: Payback Periods
EUAB: Equivalent Uniform Annual Benefit
EF: Evaluation Factor
PV: Photovoltaic
HRES: Hybrid Renewable Energy System
DG: Diesel Generator
NPC: Net Present Cost
LPSP: Loss of Power Supply Probability
AMVO: Amended Multi-Verse Optimizer
MV: Multi-Verse
AMVOA: Amended Multi-Verse Optimization Algorithm
LOA: Lion Optimization Algorithm
PIO: Pigeon-Inspired Optimization Algorithm
SDO: Supply-Demand-Based Optimization
BBO: Biogeography-Based Optimizer
EA: Evolutionary Algorithm
MGOA: Modified Grasshopper Optimization Algorithm
IGWOA: Improved Gray Wolf Optimization Algorithm
IAOA: Improved Arithmetic Optimization Algorithm
STD: Standard Deviation
BESS: The Battery Energy Storage System
HOMER: Hybrid Optimization of Multiple Electric Renewables
HESS: hybrid energy storage systems
MVOA: Original Multi-Verse Optimizer Algorithm

**Nomenclature**
$v_{rated}$: rated wind speed
$v_{cutin}$: Cut-in wind speed
$v_{couout}$: Cut-out wind speed
v: Local wind speed for the wind turbine generator
$\eta_{W}$: the wind turbine generator efficacy
$A_{W}$: the swept area
$R_{PV}^{t}$: the solar radiation
$\eta_{PV}$: PV array efficiency
$A_{PV}$: PV module area
${At}_{bat}$: the battery autonomy
$D_{l}$: the load demand
DOD: discharge depth
$\eta_{b}$: the efficiency of the battery
$\eta_{i}$: the inverter
$P_{DG}^{Out}$: the diesel generator's output power
$F_{DG}$: the fuel consumption
$A_{g}$: constant values
$B_{g}$: constant values
$F_{DG}$: the price of the fuel
$C_{R}$: the replacement costs
$C_{O\&M}$: the operating and maintenance costs
$C_{c}$: the capital cost
$C_{WT/PV}$: the wind turbine and photovoltaics' capital cost
$\beta_{WT/PV}$: initial cost
$A_{WT/PV}$: the available area
$\beta_{bat}$: the initial cost of the battery
$C_{b}$: the investment cost of the battery energy storage system
$\alpha_{bat}$: the battery's yearly operating and maintenance cost
σ: inflation rate
$N_{bat}$: the battery system's lifetime
M: the lifetime of the project
$j_{r}$: the interest rate
$\alpha_{WT/PV}$: signifies the yearly operation and maintenance costs for all components
μ: specifies the rate of escalation
$C_{O\&M,bat}$: The battery energy storage's initial operating and maintenance costs
$P_{inv}$: the rated power of the inverter
$\beta_{inv}$: the initial cost of the inverter
$\alpha_{bat}$: the inverter's yearly operating and maintenance cost
$P_{DG}$: the rated power of the DG
$\beta_{DG}$: the initial cost of the DG
$\alpha_{DG}$: the DG yearly operating and maintenance cost
$N_{DG}$: DG lifetime
$R_{DG}$: the yearly replacement cost of the DG
$P_{DG}$: DG rated power
$C_{f}$: cost of the fuel consumed value
$p_{f}$: cost of the fuel consumed value of the case study
$F_{DG}$: fuel price, fuel consumption
$P_{L}$: the load power
$E_{bat}^{miv}$: the minimum value of the battery energy in the discharge
NPC: the net present cost
CRF: the capital recovery factor
R: discount rate and the project's lifetime or duration
A: the availability factor
$P_{bat}^{t}$: the battery power
$P_{bat}^{min}$: the minimum battery state
k: constant value
RF: the percentage of Renewable energy
$P_{re}$: the sum of the renewable energy power
$C_{bat}$: the investment cost of the battery energy storage system
$P_{DG}$: the DG sum of the renewable energy power
$A_{PV}$: the photovoltaic
$A_{WT}$: the availability factor of wind turbine
$P_{WTG}$: the power produced by a wind turbine
$P_{W}$: the wind turbine's output power
$C_{O\&M,WT/PV}$: the operating and maintenance expenses

## 1 Introduction

### 1.1 Background

The demand for more effective and dependable energy distribution networks has grown as the globe continues to move toward renewable energy sources [1]. In contrast to conventional grid systems, microgrid systems have emerged as a possible solution to this issue [2]. Regional power distribution networks called Microgrids can operate separately from or in conjunction with the main electrical grid [3]. They consist of a network of interconnected power generators, such as solar cells, wind turbines, and batteries, that can generate, store, and provide electricity to a specific area [4]. They provide a consistent and ecologically friendly source of electricity, making them perfect for remote locations that are not connected to the grid and regions where the system is unreliable or prone to outages [5].

Microgrid systems are gaining popularity due to their ability to integrate renewable energy sources like wind and sunshine into the energy mix [6]. By doing so, carbon dioxide emissions can be reduced, hence reducing the impact of global warming [7]. However, several issues, such as lack of design and operation standardization and the high price of energy storage systems have hindered the deployment of microgrid networks [8]. Additionally, even though the price of clean energy has significantly declined over the past ten years, the cost of energy storage systems is still high, and investing in Microgrid systems is difficult to defend [9].

Microgrid systems are likely to be developed in the next years due to their capacity to function independently, incorporating renewable energy sources, and improving the robustness of important infrastructure assets [10]. To revolutionize the processes of energy creation, storage, and distribution, further research and development are necessary to address challenges related to consistency and cost-effectiveness [11]. One of the primary benefits of microgrid structures for storing electricity is the capacity for effectively controlling the energy provided by clean energy sources [12]. Microgrid energy storage design can reduce reliance on fossil fuels and improve Microgrid system's durability during grid outages. Additionally, it can help lessen carbon dioxide emissions and the effects of climate change [13]. The high price of energy storage systems has, however, prevented the development of Microgrid systems from incorporating energy storage [14]. Therefore, making investments in energy-storage of Microgrid systems is challenging to justify, especially in areas where the main power grid is already reliable [15].

Microgrid design for energy storage is a complex system that needs careful planning and management to operate at its best. Despite these challenges, it is anticipated that in the coming years, demand for Microgrid systems with energy storage will rise as renewable energy sources become more affordable and there is a greater need for dependable and sustainable energy storage solutions [16]. Microgrid design for energy storage is a complex system that needs careful planning and management to operate at its best. Despite these challenges, the demand for Microgrid systems with energy storage is anticipated to rise in the coming years as renewable energy sources become more affordable, and there is a greater need for dependable and sustainable energy storage solutions [17]. To overcome the issues with cost and standards, further research and development is necessary [18].

The use of optimization techniques, known as metaheuristics, allows for the resolution of challenging problems that conventional methods are unable to solve [19]. These algorithms may be used to locate the optimal solution in large search regions since they are based on natural phenomena like evolution and swarm behavior [20]. Metaheuristic approaches may be used to improve the design of Microgrids for energy storage by determining the best position for energy storage devices and renewable energy sources inside the microgrid system [21]. One of the main advantages of using metaheuristic algorithms for Microgrid design is the capacity to simultaneously address many goals, including cost reduction, reliability improvement, and reduction of greenhouse gas emissions [22].

However, due to the complex nature of the optimization problem, the use of Metaheuristic approaches for Microgrid design for energy storage is still in its infancy, and the accuracy of the results obtained using Metaheuristic algorithms may be influenced by the level of accuracy of the information being provided and the optimization variables selected [23].

As the advantages of Microgrid systems with energy storage become clearer and there is a demand for more effective and dependable energy storage solutions, it is anticipated that the usage of metaheuristic methods for microgrid design for energy storage will increase. Despite these difficulties, it is expected that Metaheuristic algorithms will be used more frequently in Microgrid design. The efficiency and dependability of Microgrid systems might be greatly increased using Metaheuristic algorithms. However, further investigation and development are required to handle the issues with complexity and standardization.

A Biofuels-integrated green power Microgrid to store electricity was optimized under uncertainty by Zheng et al. [24]. In Biomass-integrated Microgrids producing power and heat, uncertainties were assessed using predictable limited optimizing and random optimization approaches. To evaluate the planning and design of Microgrid networks utilizing BCHP, a financial Linear Programming (LP) framework with a sliding time frame was created. In Davis, California, case research was investigated for a hypothetical utility grid-connected Microgrid utilization. Based on the expected energy load profile, local climatic data, utility tariff framework, and considering technical and economic outcomes of the different Microgrid elements, the findings revealed that a BCHP/PV with battery storage combination was the greatest cost-effective design. Using Monte Carlo simulation, a density function with probabilities for the cost of electricity was created after uncertainties regarding financial and meteorological assumptions were assessed.

According to a study by Kharrich et al. [25], an improved arithmetic optimizer was used to develop the El Kharga Oasis in Egypt's Microgrid to store energy. The integrated green energy system design presented in this research includes a PV, wind farm, diesel generator, and battery system. The goal was to reduce the overall net current cost, which covers all expenses incurred throughout the project. The new method, known as IAOA, was created by updating the initial Arithmetic Optimization Algorithm(AOA) with the help of the Aquila Optimizer's (AO) leading operators. Two HRES scenarios were put out, the first of which relied on PV, wind, diesel, and battery power, and the second of which used PV, diesel, and battery power. The outcomes showed that the suggested IAOA outperforms other well-known algorithms such as the original AOA, Equilibrium Optimizer (EO), Gray Wolf Optimization (GWO), Artificial Electric Field Algorithm (AEFA), and Harris Hawks Optimization (HHO). It was acknowledged that the suggested IAOA was an effective solution for integrated green power networks.

Gomes et al. [26] researched an optimization study on a typical renewable Microgrid energy system with energy storage. In isolated Microgrids and remote regions, the challenge of developing reliable and self-sufficient renewable energy systems was amplified due to the need for grid flexibility options. One of the leading solutions to increase renewable energy usage in isolated systems was the commission of energy storage. The current study proposed a novel optimization model that sized the most cost-efficient renewable power capacity mix of an autonomous Microgrid supported by storage technologies. The proposed algorithm considered operational, technical, and land-use constraints. The problem was formulated using linear programming, was tested and scrutinized with sets of historical weather, load demand, and installation prices data, and was modeled hour-by-hour. The method was applied to Corvo, an island in the Azores archipelago, Portugal. The results showed that the proposed approach provided the optimal configuration of the renewable-based Microgrid with an LCOE (Levelized Cost of electricity) of 0.21 €/kWh, a value lower than a diesel-based alternative while ensuring minimum land area occupation. Furthermore, sensitivity analysis was also presented to examine the effect of variables on the system's LCOE and PC (present cost). The present study showed that the developed optimal sizing model could improve electricity planning and facilitate energy transition in distributed power systems.

Yee Mah et al. [27] used the P-graph method for optimizing solar electric-based Microgrids with integrated electricity storage. In this paper, a paradigm for multi-period P-graph optimization of solar Microgrids with battery-hydrogen energy storage was proposed. Results indicated that a carbon price of at least $1000 per year was needed to make a Microgrid with hybrid battery-hydrogen storage more cost-effective than traditional energy, and the optimal cost is 704,990 USD/year. The overall cost and necessary carbon price decreased to 262,334 USD/year and 300 USD/year by replacing the hydrogen storage system with grid support.

Optimized Component Design and Forward-Looking Dispatch of an Electricity Microgrid were used by Whitefoot et al. [28] for energy storage modeling. To plan for future energy storage, this research suggested adopting forward-looking optimum dispatch to improve Microgrid designs. It gave a case study of a military post that was “islanded” and had a Microgrid with both renewable and non-renewable energy sources, battery storage, and plug-in cars that could export power. Results revealed that the forward-looking method reduced expected fuel usage by 7.8 % by using storage batteries to plan for future energy shortages rather than only as a buffer for unpredictable renewable energy supplies. Investment in renewable energy technology was justifiable at gasoline costs of more than $5 per gallon ($1.32/litre), with a corresponding reduction in fuel usage of 3–30 %, according to sensitivity analysis of the best design concerning fuel price.

In this work, an optimal arrangement of a CCHP system based on the optimal selection of its parameters was proposed. Assuming the gas engine was the prime mover, the scenario was analyzed. Constrained 4E analysis was also taken into account in this case, along with fuel energy use efficacy, environmental analysis, overall energy effectiveness constraints, exergy evaluation limitations, payback periods (PB), such as exergy evaluation limitations, exergy evaluation limitations, and equivalent uniform annual benefit (EUAB). The evaluation factor (EF) was then used to select the gas engine's optimal volume for the CCHP system. An updated metaheuristic algorithm served as the foundation for optimizing the system. The final findings showed that the proposed strategy is more effective for the targeted goal.

## 2 System description

In this study, Wind, Photovoltaic (PV), Battery Energy Storage Systems, and Diesel make up a Hybrid Renewable Energy System (HRES). Modeling the system's components was required to establish the best size for each unit. Fig. (1) visually depicts the configuration of the HRES and how the various units are connected, along with thorough modeling of the preferred standalone grid architecture.

**Fig. 1:** Visual depiction of the configuration of the proposed HRES.

The modeling approach is essential for determining the system components' optimal design, taking into consideration aspects like energy consumption, the accessibility of cost-effectiveness, and renewable energy sources. It will be possible to gain a thorough knowledge of the suggested HRES and ensure that it has been designed to perform best under various circumstances by building and modeling these distinct units. To demonstrate how the HRES operates, Fig. (2) provides a block schematic of the system controller.

**Fig. 2:** Block schematic of the system controller.

The system controller's block diagram shown in Fig. (2) demonstrates how the various parts of the HRES cooperate to guarantee that the load's energy requirements are satisfied while maximizing the usage of renewable energy sources. The HRES is built to function successfully and efficiently in a variety of settings, decreasing their reliance on fossil fuels and promoting the development of an environmentally friendly energy future.

To fulfill the energy needs of the load, the system intends to generate most of its electricity from PV and wind units. A Diesel Generator (DG) will be utilized to make up for any shortfall in power if the energy produced by these units plus battery storage is not enough to fulfill the energy requirement.

On the other side, the extra electricity will be used to charge the battery when the power produced by the wind units and PV exceeds the energy requirement of the load. It makes it possible to maintain the system's readiness to fulfill energy demands, even when wind and solar energy production is low. The electricity produced by the PV and Wind Generators will be wasted once the battery has reached its maximum charging level. Yet, since the fake load consumes it, the electricity that is lost, is not wasted.

### 2.1 Wind turbine

2.2. Wind turbines are renewable energy systems that transform wind's kinetic energy into electricity. It comprises a rotor with rotating blades that spin when the wind blows and a generator that converts rotational energy into electricity. Wind turbines are frequently integrated with other renewable energy sources, such as solar panels or hydroelectric generators in HRES to create a more stable and constant supply of power. It is because Wind Turbines rely on wind availability, which fluctuates based on weather conditions. The swept area of a wind turbine, which is the area covered by the moving blades, determines its power production. The greater the swept area, the greater the amount of wind energy that can be caught and transformed into electrical energy. The power output is also affected by wind speed and air density. Wind turbines are available in a variety of sizes and may produce electricity ranging from a few kilowatts to many megawatts. The formula below may be used to calculate the power produced by a wind turbine [29] equations [[1], [2], [3], [4], [5], [6], [7], [8], [9], [10], [11], [12], [13], [14], [15], [16], [17], [18], [19], [20], [21], [22], [23], [24], [25], [26]].

(1) $$P_{WTG}=\left\{ \begin{array}{c} 0\;v<v_{ci}\\ \begin{array}{c} \frac{P_{r}\times \left(v^{3}-v_{cutin}^{3}\right)}{v_{r}^{3}-v_{cutin}^{3}}\;v_{cutin}\leq v\leq v_{rated}\\ P_{r}\;v_{rated}\leq v\leq v_{couout}\\ 0\;v>v_{couout} \end{array} \end{array}\right.$$

Where, $v_{rated}$ describes the rated wind speed, and $v_{cutin}$, $v_{couout}$, and v describe, in turn, the cut-in, cut-out, and local wind speed for the wind turbine generator. At last, the wind turbine's output power may be produced by doing the following:

(2) $$P_{W}=P_{WTG}\times A_{W}\times \eta_{w}$$

Where, $\eta_{W}$ and $A_{W}$ indicate, in turn, the wind turbine generator efficacy and the swept area.

### 2.3 Photovoltaic system

A Photovoltaic (PV) system is a type of technology that transforms solar energy into electricity. It is frequently utilized in HRES, which integrates various sources of energy to enhance reliability and effectiveness [30]. A PV system's power production is determined by various parameters, including PV module area, solar radiation, and PV array effectiveness. The quantity of sunlight that falls on the PV module is referred to as solar radiation (W/m2). The area of a PV module refers to the size of the solar panel (m2). The percentage of solar energy turned into electricity by the PV module is referred to as PV array efficiency. Shade, temperature, and the angle of the PV module concerning the sun are all elements that influence it.

The power output of a PV system can be calculated using the following formula:

(3) $$P_{PV}^{t}=R_{PV}^{t}\times \eta_{PV}\times A_{PV}$$

where, $R_{PV}^{t}$, $\eta_{PV}$, and $A_{PV}$ represent, in turn, the solar radiation, PV array efficiency, and the PV module area.

A PV system may be integrated with different technologies such as a wind turbine and hybrid energy storage systems (HESS) to produce a more reliable and effective source of electricity in an HRES.

### 2.4 Battery energy storage system

Compared to separate systems, a hybrid renewable energy system that combines photovoltaic (PV), wind turbine, and battery technologies can cut costs and enhance energy output. Approaches for calculating the cost and value contribution in capacity expansion models must be developed to appropriately estimate the market potential of wind/PV + battery systems. This covers capacity planning strategies used by utilities.

Several criteria must be examined to determine battery capacity concerning battery autonomy, load demand, inverter and battery efficiency, and depth of discharge. The battery system's capacity needs to be sufficiently big to deliver enough energy to fulfill load demand when the solar power plant fails to generate enough electricity. The battery's independence, or the amount of time it can deliver energy without being recharged, ought to be taken into account to guarantee that there is adequate energy storage capacity to fulfill load demand throughout periods of low PV energy output.

The lifespan and total capacity of the battery should also be determined by taking into consideration the depth of discharge, or the amount of energy that can be removed from the battery with no harming it. To guarantee that the system can effectively convert and store energy for later use, consideration should also be given to the inverter and battery performance. Therefore, the battery capacity can be mathematically considered as follows [31]:

(4) $$C_{bat}=\frac{D_{l}\times {At}_{bat}}{DOD\times \eta_{b}\times \eta_{i}}$$

Where, ${At}_{bat}$ specifies the battery autonomy, $D_{l}$ describes the load demand, DOD represents the discharge depth, and $\eta_{b}$ and $\eta_{i}$ describe, in turn, the efficiency of the battery and the inverter.

### 2.5 Diesel generator

When renewable energy output is minimal, a hybrid energy system might incorporate a diesel generator to supply backup power to the load. It is required to take into account the diesel generator's fuel consumption, output power, and linear fuel consumption to calculate its rated power in a hybrid system. The output power of a diesel generator—the highest amount of electricity it can deliver to the load—determines its rated power. The diesel generator's fuel consumption depends on both its output power and generator performance. The quantity of fuel spent per unit of electrical energy produced by the diesel generator is referred to as linear fuel consumption.

It is required to balance the diesel generator's output power with the load's power demand during low renewable energy generation times to determine the diesel generator's rated power in a hybrid energy system. Understanding the load profile, which details the electrical demand of the load across time, is necessary for this. The diesel generator's rated output must be adequate to handle the load's peak power requirements while reducing fuel use and pollutants.

In simple terms, the output power of the diesel generator is balanced with the power demand of the load during times of low renewable energy production to figure out the rated power of the diesel generator in an HRES. When choosing a diesel generator for a hybrid system, it is necessary to take fuel consumption and linear fuel consumption into account. The formula for calculating the diesel-rated power is as follows:

(5) $$P_{DG}=\frac{F_{DG}-A_{g}\times P_{DG}^{Out}}{B_{g}}$$

Where, $P_{DG}^{Out}$ specifies the diesel generator's output power, $F_{DG}$ signifies the fuel consumption, and $A_{g}$ and $B_{g}$ describe, in turn, two constant values.

## 3 Optimization purpose

### 3.1 Objective function

An optimization problem's target must be attained according to an objective function, which is a mathematical expression. Objective functions can be utilized to optimize the design and operation of Microgrids with energy storage devices for effective and sustainable energy management. Therefore, objective functions can offer useful insights and techniques for optimizing the operation and design of Microgrids by taking a variety of aspects into account, such as renewable energy sources, energy demand, and energy storage systems.

#### 3.1.1 Net present cost (NPC)

By predicting the timing and cost of a project or investment and discounting those expenses to their present value utilizing a discount rate, Net Present Cost (NPC) may be estimated. The NPC would be the total of the cost's current values. The NPC might describe the present value of expenditures related to a project or investment, which could be determined using methods.

The NPC stands for an economic element, which is regarded as the study's objective function. The goal of this study is to reduce the total NPC expenses during the project. The formula for calculating the NPC is:

(6) $$NPC=F_{DG}+C_{R}+C_{O\&M}+C_{c}$$

where, $F_{DG}$ describes the price of the fuel, and $C_{R}$, $C_{O\&M}$, and $C_{c}$ represent, in turn, the replacement costs, the operating and maintenance costs, and the capital cost.

Expenditures of wind turbine and Photovoltaic costs for wind turbine and Photovoltaic are modeled similarly. Concerning their initial cost and the available area, the wind turbine and Photovoltaics’ capital cost ($C_{WT/PV}$) is computed [35].

(7) $$C_{WT/PV}=A_{WT/PV}\times \beta_{WT/PV}$$

Where, initial cost and the available area are defined by $\beta_{WT/PV}$ and $A_{WT/PV}$, respectively. The operating and maintenance expenses are determined as follows:

(8) $$C_{O\&M,WT/PV}=\alpha_{WT/PV}\times A_{WT/PV}\times {\sum_{j}\left(\frac{1+\mu }{1+j_{r}}\right)}^{j}$$

Where, $\alpha_{WT/PV}$ signifies the yearly operation and maintenance costs for all components, μ specifies the rate of escalation, $j_{r}$ describes the interest rate, and j=1,2,…,M such that M specifies the lifetime of the project. Since the project lifespan and the Photovoltaic, or wind turbine lifetime are the same, the replacement costs are zero.

The battery energy storage's initial operating and maintenance costs can be achieved based on the following equations:

(9) $$C_{battery}=\beta_{bat}\times C_{b}$$

(10) $$C_{O\&M,bat}=\alpha_{bat}\times C_{b}\times {\sum_{j}\left(\frac{1+\mu }{1+\sigma }\right)}^{\left(j-1\right)N_{bat}}$$

Where, $\beta_{bat}$ describes the initial cost of the battery, $C_{b}$ specifies the investment cost of the battery energy storage system, $\alpha_{bat}$ describes the battery's yearly operating and maintenance cost, σ signifies the inflation rate, and $N_{bat}$ specifies lifetime of the battery system.

As shown in Ref. [32], the operating and maintenance cost and investment costs of the inverter can be achieved by the following equations:

(11) $$C_{inv}=\beta_{inv}\times P_{inv}$$

(12) $$C_{O\&M,inv}=\alpha_{inv}\times {\sum_{j}\left(\frac{1+\mu }{1+j_{r}}\right)}^{j}$$

Where, $P_{inv}$ , $\beta_{inv}$, and $\alpha_{bat}\text{,}$ describe, in turn, the rated power of the inverter, the initial cost of the inverter, and the inverter's yearly operating and maintenance cost.

Finally, the Diesel Generator's cost can be achieved as follows [32]:

(13) $$C_{DG}=\beta_{DG}\times P_{DG}$$

(14) $$C_{O\&M,DG}=\alpha_{DG}\times N_{DG}\times {\sum_{j}\left(\frac{1+\mu }{1+j_{r}}\right)}^{j}$$

(15) $$R_{Diesel}=R_{DG}\times P_{DG}\times {\sum_{j=7,14,\ldots }\left(\frac{1+\sigma }{1+j_{r}}\right)}^{j}$$

(16) $$C_{f}^{t}=p_{f}\times F_{DG}$$

(17) $$FC_{\text{DG}}=\sum_{t=1}^{8760}C_{f}\times \sum_{j=1}^{M}{\left(\frac{1+\sigma }{1+j_{r}}\right)}^{j}$$

Where, $P_{DG}$ , $\beta_{DG}$, $\alpha_{DG}\text{,}$ $N_{DG}$, $R_{DG}$, $P_{DG}$, $C_{f}$, $p_{f}$, and $F_{DG}$, describe, in turn, the rated power of the DG, the initial cost of the DG, the DG yearly operating and maintenance cost, DG lifetime, the yearly replacement cost of the DG, DG rated power, cost of the fuel consumed value, cost of the fuel consumed value of the case study, fuel price, and fuel consumption.

#### 3.1.2 LPSP index

The Loss of Power Supply Probability (LPSP) is a measure of the risk that a power supply may fail or be interrupted, causing a system or device to lose power. It is commonly represented as a percentage or likelihood over a particular period. This possibility can be influenced by a variety of factors, including power supply quality and dependability, ambient conditions, and maintenance procedures. A higher LPSP implies a larger possibility of a power failure and may necessitate additional steps to assure system dependability and uptime. In this study, the LPSP index is used as a part of the objective function as follows:

(18) $$LPSP=\frac{\sum_{t=1}^{8760}\left[P_{L}^{t}+E_{bat}^{\min}-P_{WT}^{t}-P_{PV}^{t}-P_{DG}^{O,t}\right]}{\sum_{t=1}^{8760}P_{L}^{t}}$$

Where, $P_{L}$ signifies the load power, and $E_{bat}^{miv}$ describes the minimum value of the battery energy in discharge.

#### 3.1.3 LCOE index

The term Levelized Cost of Power (LCOE) refers to the average cost of producing power from a certain energy source during the lifetime of the Microgrid. It is a cost-benefit analysis that considers all expenses connected with the construction and operation of a power plant, including initial capital costs, fuel prices, maintenance costs, and the cost of financing the project. The LCOE index compares the cost of producing electricity from various energy sources. This index can be achieved by the following equation:

(19) $$LCOE=\frac{NPC\times CRF}{\sum_{t=1}^{8760}P_{L}^{t}}$$

Where, NPC describes the net present cost, and CRF describes the capital recovery factor and is achieved as follows:

(20) $$CRF=\frac{j_{r}\times {\left(1+j_{r}\right)}^{R}}{{\left(1+j_{r}\right)}^{R}-1}$$

Where, $j_{r}$ and R describe the interest rate or discount rate and the project's lifetime or duration, respectively.

#### 3.1.4 Availability index

The availability factor (A) is thought to be an indication of customer satisfaction; it assesses the Microgrid's capacity to convert total energy to load charge. The availability is computed as follows:

(21) $$A=1-\frac{DMN}{\sum_{t=1}^{8760}P_{L}^{t}}$$

(22) $$DMN=P_{bat}^{\min}-P_{bat}^{t}-k\left(t\right)\times \left[P_{WT}^{t}+P_{PV}^{t}+P_{DG}^{O,t}-P_{L}^{t}\right]$$

Where, $P_{bat}^{t}$ describes the battery power, $P_{bat}^{\min}$ specifies the minimum battery state, k is a constant value that the load is not fulfilled, when k=1, else, k=0.

#### 3.1.5 RE index

Renewable Energy (RE) is measured to assess the percentage of renewable energy that has permeated the Microgrid system. The RE is written as follows:

(23) $$RF=1-\frac{\sum_{t=1}^{8760}P_{DG}^{O,t}}{\sum_{t=1}^{8760}P_{re}^{t}}$$

Where, $P_{re}$ signifies the sum of the renewable energy power.

### 3.2 Constraints

Constraints are restrictions or criteria that must be met during Microgrid system optimization or control. The performance of the Microgrid may be enhanced by applying suitable limitations in terms of several objectives including dependability, efficiency, and sustainability. Here, 8 constraints have been utilized for the optimization.

(24) $$\left[\begin{array}{c} 0\\ 0\\ 0\\ 0 \end{array}\right]\leq \left[\begin{array}{c} A_{PV}\\ A_{WT}\\ C_{bat}\\ P_{DG} \end{array}\right]\leq \left[\begin{array}{c} A_{PV}^{\max}\\ A_{WT}^{\max}\\ C_{bat}^{\max}\\ P_{DG}^{\max} \end{array}\right]$$

Where, $C_{bat}$ signifies the investment cost of the battery energy storage system, $P_{DG}$ specifies the DG sum of the renewable energy power, and $A_{PV}$ and $A_{WT}$ represent, in turn, the availability factor of the Photovoltaic and wind turbine, all of which are fully illustrated below:

(25) $$\left[\begin{array}{c} A^{\min}\\ {At}_{bat}^{\min}\\ RE^{\min}\\ LPSP^{\min} \end{array}\right]\leq \left[\begin{array}{c} A\\ {At}_{bat}\\ RE\\ LPSP \end{array}\right]$$

Where, A describes the availability factor, RE signifies the percentage of renewable energy, and LPSP defines the Loss of Power Supply Probability.

## 4 Amended multi-verse optimizer (AMVO)

### 4.1 Motivation

Based on the theory of the big bang, a massive explosion caused the start of our universe. Recently, the theory of Multi-verse (MV) has become well-known among scientists. This theory expresses that more than one big bang is involved in the universe's appearance, and it does refer to the other universes' existence which interact and may crash with each other. Moreover, this theory proposes that various laws of physics may exist in every universe.

For expressing the MVO motivation, three key concepts of the MV have been chosen: black holes, white, and wormholes. Although a white hole has no longer been observed in our universe, physicists believe that the white hole could be the big bang as the key element in the universe's appearance. In the cyclic mode of the MV theory, there is also an idea that white holes or big bangs have been shaped in a location where the crashes happen amid the parallel universes. In marked contrast, the behavior of black holes is different from white ones, and they are frequently seen. These holes absorb everything, i.e., light rays with their extraordinary force of gravity. The holes that make a connection amid various sections of a universe are wormholes. These holes perform as tunnels of space/time travel, whereby everything is capable of traveling immediately from one corner of a universe to the other parts or from one universe to the others. Fig. (3 (A – C)) demonstrates the model of these three key concepts of the MV theory.

**Fig. 3:** Model of 3 key concepts: (A) Black hole, (B) white hole, and (C)wormhole.

All universes have a specific rate of inflation (named eternal); this rate provides the expansion of a universe through space. In each universe, the velocity of inflation is vital when it comes to forming stars, asteroids, planets, laws of physics, life suitability, white, black, and wormholes. In one cyclic model of multi-verse, there is an idea that there is an interaction among multiple universes by black, white, and wormholes to reach a steady condition. It expresses the main motivation of the MVO that has been simulated mathematically in the following section.

### 4.2 Multi-verse method of optimization

The search space is split into two phases of exploitation and exploration by a population-based optimizer. In this work, the concept of black-and-white holes has been utilized for exploring solution spaces via MVO. The wormholes, however, help the offered method in exploiting the solution area. Every solution has been assumed analogous to a specific universe, and every parameter over the search space is an item in that particular universe. Furthermore, every result is considered a rate of inflation, which is correlated to the solution cost function amount. In this article, the term time is also used instead of iteration because it has been a usual term in cosmology and MV theory. Throughout the process of optimizing, the below principles have been applied to the MVO universes:

1. The upper ratio of inflation, the upper possibility of white hole existence.
2. The upper ratio of inflation, the lower possibility of black hole existence.
3. Universes with an upper ratio of inflation tend to conduct items through white holes.
4. Universes with lower ratios of inflation tend to take more items through black holes.
5. The items of the total universes might confront random motions towards the finest universe by wormholes irrespective of the ratio of inflation.

The items have been permitted to make movements among diverse universes with the aim of tunnels that are black or white holes. Whenever a black or white tunnel has been settled between two universes, it is considered that white holes exist in the universe, which has a high ratio of inflation. On the other hand, it has been considered that there is a black hole in the universe that has a less ratio of inflation. Then, all items have been transferred from the source universe (white holes) to the destination one (black holes). Such a mechanism does provide a fertile ground for the universes to exchange items easily. For improving the universes’ inflation ratio, the universes with a higher inflation rate are considered to have higher chances of owing white holes. In marked contrast, the universes with a lower inflation ratio have higher chances of taking black holes. Thus, items are likely to be transferred from a high-inflation-ratio universe to a universe that has a lower ratio of inflation. Such a likeness can assure the improvement of the mean inflation ratio for all universes through epochs.

For Modeling the tunnels of black or white holes and exchanging the universes’ items based on mathematics, a mechanism of the roulette wheel was utilized. Over each epoch, the universes have been sorted based on their rate of inflation. Then, using the roulette wheel, one of the rates is chosen for owing a white hole. To implement this process, the below steps have been applied. Considering that:

(26) $$U=\left[\begin{array}{ccc} y_{1}^{1} & \cdots & y_{1}^{d}\\ \vdots & \ddots & \vdots \\ y_{n}^{1} & \cdots & y_{n}^{d} \end{array}\right]$$

Here, the parameters' number is illustrated by d (variables' quantity), and the universes' number is demonstrated by n (candidate results):

(27) $$y_{j}^{i}=\left\{ \begin{array}{c} y_{k}^{i}\;r1<NI\left(Ui\right)\\ y_{j}^{i}\;r1\geq NI\left(Ui\right) \end{array}\right.$$

Where, Ui and NI(Ui) are the indication of the universe i and its normalized ratio of inflation, respectively. $y_{j}^{i}$ and $y_{k}^{i}$ signifies the parameters i in the universe i and k, and r1 illustrates a randomly chosen amount that varies from zero to one.

Regarding Eq. (27), the roulette wheel has been implemented for choosing and determining the white holes. The lower rate of inflation illustrates the more and more possibility of items’ distribution through tunnels of black or white holes. It is imperative to note that –NI ought to be converted to NI for the problems of maximization. The process of exploration could be ensured the utilizing this mechanism until the universes have been needed to exchange items and encounter quick alterations for exploration of the solution area.

Based on the mentioned mechanism, the items are exchanged between the universes without any trace of disorders. For maintaining the variety of universes and accomplishing the phase of exploitation, all universes have been assumed to have wormholes for transporting their items over the solution space on a random basis. It might be seen that the wormholes alter the universes’ items on a random basis without assuming their rates of inflation. For providing local alterations for every universe and making a higher likelihood of improvement in the rate of inflation based on wormholes, tunnels of wormhole tunnels are assumed to be set amid a universe and the finest one. The mathematical model of the mentioned process is illustrated below equations [[28], [29], [30], [31], [32], [33], [34]]:

(28) $$y_{j}^{i}=\left\{ \begin{array}{cc} \left\{ \begin{array}{cc} Y_{i}+TSR\times \left(\left({hl}_{i}-{ll}_{i}\right)\times r4+{ll}_{i}\right) & r3<\frac{1}{2}\\ Y_{i}-TSR\times \left(\left({hl}_{i}-{ll}_{i}\right)\times r4+{ll}_{i}\right) & r3\geq \frac{1}{2} \end{array}\right. & r2<WPP\\ y_{j}^{i} & r2\geq WPP \end{array}\right.$$

Where, $Y_{i}$ does illustrate the parameter i for the finest universe, TSR and WPP are coefficients, ${ll}_{i}$ and ${hl}_{i}$ demonstrate the lowest and highest limitations of the parameter i, $y_{j}^{i}$ does signify the parameter i from the universe j, and r4, r3, and r2 demonstrate random values varying from zero to one.

Two key coefficients exist: WPP and TSR which stand for the Possibility of Wormhole Presence and Rate of Traveling Space in universes. For highlighting the phase of exploitation in the process of optimizing, there is a need for the linear escalation of WPP in each epoch. TSR does signify the rate of distance that an item could be moved from one position to another via a wormhole over the finest universe. Over the finest universe, TSR experiences an upward trend over the epochs for gaining far more exact local search or phase of exploitation. The mathematical equation for both WPP and TSR can be expressed as below:

(29) $$WPP=\mathrm{MIN}+t\times \left(\frac{\mathrm{MAX}-\mathrm{MIN}}{t_{\max}}\right)$$

(30) TSR=1−t1qtmax1/q

Where, MAX and MIN are the maximum and minimum amounts which are 1 and $\frac{1}{5}$ in this work. $t_{\max}$ and t indicate the max and existing epochs. The accuracy of exploitation in this work is defined by q that is assumed to be six through each epoch. Whenever q is high, the phase of exploitation is accurate, and it happens sooner. It is imperative to note that TSR and WPP could be assumed constants; it is recommended; however, adaptive amounts are considered for both coefficients based on the outcomes of this article.

### 4.3 Amended multi-verse optimization algorithm (AMVOA)

In this study, two improvement mechanisms are used for resolving the mentioned issues with the multi-verse optimizer, a newly introduced metaheuristic algorithm that can be used for various objectives. However, the multi-verse optimizer demonstrates well outcomes for solving in multiple applications, but it sometimes has unsuitable results due to premature convergence and local optimum outcomes.

It is clear from the results of the multi-verse optimizer's finding process that each candidate should be prospective at first, and that a local search must then be conducted to improve the people's quality. To alter the model update, assume a weight to do this. This is expressed as follows:

(31) $$y_{j}^{i}=\left\{ \begin{array}{cc} \left\{ \begin{array}{cc} Y_{i}+TSR\times \left(\left({hl}_{i}-{ll}_{i}\right)\times w+{ll}_{i}\right) & r3<\frac{1}{2}\\ Y_{i}-TSR\times \left(\left({hl}_{i}-{ll}_{i}\right)\times w+{ll}_{i}\right) & r3\geq \frac{1}{2} \end{array}\right. & r2<WPP\\ y_{j}^{i} & r2\geq WPP \end{array}\right.$$

Such that

(32) $$w=\left\{ \begin{array}{c} \left(\frac{f\left(X_{best}\right)}{f\left(X_{worst}\right)}\right),if\;f\left(X_{worst}\right)\neq 0\\ 1,o.w. \end{array}\right.$$

where the worst and greatest values of the cost function, respectively, are denoted by $f\left(X_{worst}\right)$ and $f\left(X_{best}\right)$. The difference between the best and worst solutions has been decreasing progressively, and the weight's value is a self-adaptive weighting that grows gradually. The balance between exploitation and exploration is improved as a result. The algorithm's parameters are lowered by this feature.

Applying a chaotic process is the second development. With this change, the best possible solution quality will be maintained throughout the iterations. The best solution in the process has a big impact on how well the other people are controlled. While occasionally, both local and global best solutions are equally effective. This problem results in early convergence occasionally. Using a chaotic mechanism is one appropriate way to handle this metaheuristics problem.

This method offers an ergodic and random outcome to change the solution's quality by creating some new solutions. The logistic map has been used in this investigation. Here, we used this mechanism to update $r_{2}$ and $r_{3}$ in the next iterations. It can be applied as follows:

(33) $$r_{2}\left(t+1\right)=\left[y_{best}-y_{m}\right]\times \alpha -y^{i+1}+\left(\left(H_{B}-L_{B}\right)\times y^{i+1}+L_{B}\right)\times \delta$$

where,

(34) $$y_{m+1}=4y_{m}\left(1-y_{m}\right)$$

where, $L_{B}$ and $H_{B}$ describe, in turn, the lower and the higher bounds, α and δ are the exploitation elements fixed to 0.01, $y_{m}$ describes the $m^{th}$ iteration value, and $y_{0}$ specifies an initial value that is randomly spread in the range 0 and 1.

### 4.4 Algorithm assessment

The usefulness of the suggested Amended multi-verse optimization algorithm in locating the best solution to the optimization issues in this portion of the investigation has been demonstrated. The main objective is to showcase the efficacy of the proposed Amended Multi-Verse Optimization Algorithm in efficiently solving optimization problems within this specific part of our study. To achieve this, experiments involving two Unimodal and two Multimodal benchmark problems were conducted. Through these experiments, we aimed to demonstrate the algorithm's effectiveness in finding the optimal solutions. Two Unimodal and two Multimodal Basic issues are experimented with to achieve this. The main goal was to evaluate whether the Amended multi-verse optimization method could offer these issues the best possible solutions.

For algorithm verification of the indicated Amended multi-verse optimization algorithm, four other metaheuristics from the literature, including the Lion optimization algorithm (LOA) [33], Pigeon-inspired Optimization Algorithm (PIO) [34], Supply-Demand-Based Optimization (SDO) [35], and Biogeography-Based Optimizer (BBO) [36] have been utilized. All the test functions employed in this study were meant to be minimized. The alternate settings of the optimizers are provided in Table 1.

**Table 1:** Alternate settings of the optimizers.

Algorithm	Variable	value			
LOA [33]	Number of prides	5	PIO [34]	Number of Pigeons	200
	Percent of nomad lions	0.3		Space dimension	20
	Roaming percent	0.4		Map and compass factor	0.2
	Mutation probability	0.1		Map and compass operation limit	150
	Sex rate	0.85		Landmark operation limit	200
	Mating probability	0.4		Inertia factor (w)	1
	Immigrate rate	0.5		Self-confidence factor ($c_{1}$)	1.2
BBO [36]	Habitat modification probability	1		Swarm confidence factor ($c_{2}$)	1.2
	Immigration probability bounds per gene	[0,1]	SDO [35]	MaxIteration	200
	Step size for numerical integration of probabilities	1		MarketSize	40
	Max immigration (I) and Max emigration (E)	1		FunIndex	1
	Mutation probability	0.005			

The variables of the suggested method were established empirically, especially for the specified issue, and might vary in different problems. To evaluate the efficacy of the suggested AMVOA approach, we tested it on the “CEC-BC-2017 test suite”, which is a standard benchmark system. The assessment was done on ten odd benchmark functions, with decision variable restrictions between −100 and 100. To guarantee a fair comparison with different algorithms. The population size and maximum iteration for all algorithms are set, in turn, 50 and 200.

Table 2 offers a comparison of the suggested Amended Multi-Verse Optimization Algorithm with different metaheuristics that have been applied to the CEC-BC-2017 test suite. By comparing the outcomes of these algorithms, it has been hoped to illustrate the better efficiency of the Amended multi-verse optimization algorithm in addressing global optimization issues. This work consequently gives proof of the potential of the Amended multi-verse optimization algorithm as a useful tool for tackling a wide range of real-world optimization issues.

**Table 2:** Comparison between the suggested AMVOA proposed and other metaheuristics utilized in the CEC-BC-2017 test suite.

Benchmark		AMVOA	LOA [33]	BBO [36]	PIO [34]	SDO [35]
f1	AVG	0.00	4.48	4.21	3.59	3.21
	STD	0.00	3.75	3.93	2.82	2.79
f2	AVG	0.21	4.76	4.29	4.06	3.98
	STD	0.15	4.28	3.84	3.78	2.83
f3	AVG	0.00	5.59e-3	7.68e-3	4.57e-4	6.73e-4
	STD	0.00	4.63e-4	5.21e-4	6.28e-5	8.46e-5
f4	AVG	0.00	0.00	4.39e-6	2.97e-6	1.37e-7
	STD	0.00	0.00	9.93e-6	8.84e-6	7.29e-7
F5	AVG	0.00	2.98	1.93	1.46	1.23
	STD	0.00	2.63	1.74	1.32	1.05
F6	AVG	0.05	1.75	1.66	1.52	1.38
	STD	0.01	1.53	1.39	1.21	1.12
F7	AVG	0.07	5.38	5.29	4.86	3.79
	STD	0.02	4.64	4.89	4.35	3.54
F8	AVG	0.00	0.64	0.71	0.97	1.05
	STD	0.00	0.51	0.62	0.75	0.92
F9	AVG	0.00	0.00	1.49	1.37	1.22
	STD	0.00	0.00	1.34	1.25	1.13
F10	AVG	0.00	1.45	1.39	1.26	2.13
	STD	0.00	1.34	1.28	1.15	1.68

Based on the findings shown in Table 2, the proposed AMVOA attained the maximum degree of accuracy in solving the CEC benchmark functions. This conclusion implies that the suggested methodology is more efficient than the other compared strategies. Additionally, the standard deviation (STD) value of the suggested technique is one of the lowest among the studied methods, which shows greater dependability in addressing optimization issues across several runs. The decreased standard deviation value of the suggested method in contrast to previous techniques, demonstrates its improved reliability in providing consistent and accurate findings over different runs.

The result is especially relevant as it suggests that the suggested strategy is less sensitive to alterations in the beginning circumstances or other factors that might impact the optimization process. As a result, these findings illustrate the usefulness of the proposed AMVOA in addressing global optimization issues and its potential to be implemented in many real-world settings. The excellent accuracy and dependability of the suggested approach make it a viable tool for tackling a wide range of optimization problems.

## 5 Simulation results

### 5.1 The case study under analysis

The HRES in this study uses the Serakhs area. Serakhs is an oasis city located in the Ahal Province of Turkmenistan, situated at latitude 36°31′ North and longitude 61°12′ East at an altitude of 285 m above sea level. It is one of the oases of the historic Silk Road sitting between Merv to the east and Mashhad to the west. The location of the Serakhs area is indicated in Fig. (4).

**Fig. 4:** Satellite images of the Serakhs area retrieved from Google Maps.

Fig. (5) and Fig. (6) show the load and the meteorological conditions (see Fig. 9). The statement implies that there are 6 separate figures, numbered from Fig. (5) to Fig. (10), that exhibit information regarding the load and weather conditions. These graphics possibly illustrate visual illustrations of data linked to the electrical load on a system and the meteorological conditions that impact it. The load refers to the quantity of electrical power that is being utilized by the system at a given time. This information may be used to examine the performance and efficiency of the system, as well as to detect periods of high or low demand that can be utilized to improve the operation of the system. Fig. (5) describes the profile of the load demand for one year.

**Fig. 5:** The profile of the load demand for one year.

**Fig. 6:** Metrological data for (A) PV radiation, (B) wind speed data, (C) temperature data, (D) pressure, and (E) air density.

Meteorological conditions relate to the meteorological conditions that impact the functioning of the system, such as humidity, temperature, wind speed, and sun radiation. These circumstances can have a considerable influence on the operation of renewable energy systems such as solar panels and wind turbines, as well as on the effectiveness of cooling and heating systems. Fig. (6 (A – E)) to Fig. (10) illustrate the meteorological conditions.

### 5.2 Simulations

The HRES design refers to the design of hybrid renewable energy systems that integrate multiple renewable energy sources to satisfy energy demands. The HOMER software is a tool for developing and enhancing hybrid renewable energy systems design. It includes optimization and sensitivity techniques that help to assess design possibilities simpler. The simulation operation results in a specific model configuration, whereas the optimization procedure chooses the ideal model arrangement [37]. Nevertheless, there are limits to utilizing HOMER software or related tools like HOGA for HRES design. For instance, the program demands the user to precisely input all relevant information, like resource availability and energy consumption. Furthermore, it does not give a full design solution for complex systems requiring multiple goals to be satisfied.

In recent years, various methodologies based on metaheuristics, on the other hand, provide significant benefits over classic software tools like HOMER for HRES design. These approaches can evaluate vast datasets and produce reliable predictions and suggestions, which makes them suited for complicated systems. They may additionally benefit from prior experiences and adapt to new settings, which makes them excellent for tackling new design difficulties. The metaheuristics-based approaches can also assist in decreasing human mistakes and bias, leading to more optimum and cost-effective designs. In summary, whereas traditional software tools like HOMER have limits for HRES design, metaheuristics-based solutions provide advantages such as scalability, cost-effectiveness, and accuracy.

The present study introduces a new modified metaheuristic-based technique called an Amended Multi-Verse Optimizer for the optimal design of the studied HRES. The proposed AMVOA is utilized to create the HRES based on two different configurations to demonstrate its usefulness in resolving complicated problems. One configuration includes a photovoltaic, wind turbine, diesel generator, and battery energy storage system, and the other is just based on a photovoltaic, diesel generator, and battery energy storage system. The main purpose of the study is to provide electricity to a home in the Serakhs area.

#### 5.2.1 Scenario 1: wind/PV/DG/BESS

The first assessed arrangement is the Wind/PV/DG/BESS structure, which benefits from the complementarity of the wind turbine and Photovoltaic resources. In comparison, five algorithms, including the Evolutionary Algorithm (EA) [38], Modified Grasshopper Optimization Algorithm (MGOA) [39], Improved Gray Wolf Optimization Algorithm (IGWOA) [40], Improved Arithmetic Optimization Algorithm (IAOA) [25], and the original MVOA were utilized. The suggested AMVOA yields the optimum project investment in Fig. (7 (A – B)).

**Fig. 7:** Optimal results of the HRES based on Wind, PV, DG, and BESS structure for (A) NPC,RF, and Availability, and for (B) LCOE and LPSP.

The optimal results from the AMVOA include an NPC (Net Present Cost) of 299,010 dollars, which is equivalent to an energy cost of 0.2309 dollars per kilowatt-hour. It indicates that the proposed technique has successfully minimized the energy system's overall cost while maintaining its reliability and efficiency. Furthermore, the proposed technique has been able to meet the defined limitations, such as a 5.22 % LPSP (Loss of Power Supply Probability), which is a measure of the system's reliability. The high electricity availability of 99.83 % indicates that the system is capable of providing power to consumers most of the time. Additionally, the renewable portion of the energy system is 84.86 %, indicating that the proposed technique has successfully incorporated a significant amount of renewable energy sources into the system. Fig. (8) presents the optimal sizing of the HRES based on Wind, PV, DG, and BESS structure.

**Fig. 8:** Optimal sizing of the HRES based on Wind, PV, DG, and BESS structure.

As can be observed, Fig. (8) demonstrates that the optimal Photovoltaic area of 155.8 $m^{2}$ is determined by the sizing algorithm based on factors such as available rooftop or ground space, solar irradiance levels, and energy demand. A swept wind area of 263.4 $m^{2}$ is required for wind turbines to capture wind energy effectively. Factors such as wind speed, direction, and site characteristics should be considered to determine the appropriateness of this area. A storage capacity of 12.89 kWh is suggested for the Battery Energy Storage System (BESS) of the HRES. Evaluating the storage capacity is crucial to meet energy demand during low renewable energy generation or high load demand periods. Factors such as desired autonomy time and depth of discharge should be considered. The nominal diesel power of 17.89 kW represents the rated power of the Diesel Generator (DG) component in the HRES. The sizing of the DG should be based on the energy deficit that cannot be covered by renewable sources or storage, fuel availability, cost, and environmental impacts. In assessing these results, it is essential to consider the specific requirements, constraints, and objectives of the HRES system, such as load demand, renewable resource availability, system efficiency goals, and budgetary considerations. Comparing these results with alternative sizing approaches or established industry standards can evaluate their efficiency, cost-effectiveness, and feasibility in real-world applications.

Fig. (9) shows an overview of all algorithms' convergence curve findings, and it is clear from the figure that the AMVOA provides a better convergence solution.

**Fig. 9:** Convergence curve of the studied algorithms for the Wind, PV, DG, and BESS structure.

**Fig. 10:** Power output for the Wind, PV, DG, and BESS structure: (A) BESS, (B) DG, (C) PV, and (D) WT.

Fig. 10 (A – D) depicts the output power of all algorithms during 1 day, ranging from 1000 to 1024 h.

According to Fig. (10), the output power curves of the Wind, PV, DG, and BESS structure are efficiently handled, the Photovoltaic is the pillar system, and the BESS is employed to accomplish economic and technological customer satisfaction.

#### 5.2.2 Scenario 2: PV, DG, and BESS

The second assessed arrangement is the PV, DG, and BESS structure, which benefits from the complementarity of the Photovoltaic resources. The suggested AMVOA yields the optimum project investment in Fig. (11 (A – B)).

**Fig. 11:** Optimal results of the HRES based on PV, DG, and BESS structure for (A) NPC,RF, and Availability, and for (B) LCOE and LPSP.

The findings from Fig. (11) reveal that the most effective investment plan is determined employing the modified AMVOA method at a cost of 333,800 $, comparing to an energy cost of 0.3451 $/kWh. It designates that the suggested method has been effective in minimizing the total cost of the energy system while maintaining its reliability and efficiency. Fig. (12) presents the optimal sizing of the HRES based on PV, DG, and BESS structure.

**Fig. 12:** Optimal sizing of the HRES based on PV/DG/BESS structure.

As can be observed from Fig. (12), the optimal sizing of a Hydrogen Energy Storage System (HRES) is determined by the optimal combination of PV, DG, and BESS structures. The optimal Photovoltaic area is 243.8 $m^{2}$, which is suitable for capturing efficient solar energy. The diesel capacity is 18.19 kW, which is the required power capacity for the Diesel Generator (DG) component in the HRES. The DG should be based on factors such as load demand, energy deficit, fuel availability, cost, and environmental considerations. The optimal design does not require a Battery Energy Storage System (BESS), indicating that the combination of PV and DG is sufficient without additional energy storage.

However, the absence of a BESS may impact the system's ability to manage intermittencies and address fluctuations in load demand. Assessing the trade-off between the cost of implementing a BESS and its benefits in terms of stability and reliability is necessary.

To analyze these results, it is essential to consider specific requirements, constraints, and objectives of the HRES system, such as load demand, renewable resource availability, efficiency goals, and budgetary considerations. Comparing these results with alternative sizing approaches or industry standards is also valuable for evaluating their efficiency, cost-effectiveness, and feasibility in real-world applications.

A comprehensive analysis should be conducted to assess the reliability and performance of the proposed HRES configuration without a BESS in managing renewable energy intermittencies and meeting load demand consistently. It is crucial to consider scenarios such as low solar irradiance, high load demand, and fuel availability limitations to evaluate the robustness and practicality of the sizing solution obtained by the AMVOA algorithm. Fig. (13) shows an overview of findings of all algorithms' convergence curve, and it is clear from the figure that the AMVOA provides a better convergence solution.

**Fig. 13:** Convergence curve of the studied algorithms for the PV, DG, and BESS structure.

Fig. (14) depicts daily output power from 1000 to 1024 h to help understand power management behavior. The following figures depict the amount of power management that has been employed.

According to Fig. (14), the output power curves of the PV, DG, and BESS structure are efficiently handled, the Photovoltaic is the pillar system, and the BESS is employed to accomplish economic and technological customer satisfaction. We concluded from the findings that the suggested approach's performance is promising due to the provided improvements, which aid the traditional method in identifying new answers and search regions. Furthermore, it may switch between search procedures to identify better results and avoid complications with searching.

**Fig. 14:** Power output for the PV, DG, and BESS structure: (A) BESS, (B) DG, (C) PV, and (D) WT.

The research work provides information on the shortcomings of various optimization methods, including the Evolutionary Algorithm (EA), Modified Grasshopper Optimization Algorithm (MGOA), Improved Gray Wolf Optimization Algorithm (IGWOA), Improved Arithmetic Optimization Algorithm (IAOA), and Original Multi-Verse Optimizer Algorithm (MVOA). These methods may suffer from slow convergence rates, premature convergence, and local optima, which can hinder the algorithm's ability to reach an optimal solution. Assessing the improvements made in these algorithms is crucial to understand their limitations.

The modified MGOA may address some limitations of the original algorithm, but it is essential to assess whether these modifications improve solution quality and convergence speed. The improved IGWOA, inspired by the social hierarchy and hunting behavior of gray wolves, has been improved. However, it is crucial to evaluate whether these improvements effectively improve convergence and solution quality compared to the original algorithm.

In conclusion, the proposed algorithm was chosen based on several grounds demonstrating its suitability for addressing the specific challenges and objectives of the Microgrid optimization problem. Some logical reasons for the selection are given in the following. The algorithm exhibits robust performance in prior research, showcasing encouraging outcomes in the optimization of energy storage arrangements, enhancement of system efficiency, and attainment of goals such as cost reduction and integration of renewable sources. The proposed approach exhibits scalability and flexibility, incorporates considerations for uncertainty, and achieves a harmonious trade-off between computing complexity and solution quality. The algorithm benefits from an active research community, comprehensive documentation, and robust support, providing access to valuable resources and expert help. The validation and resilience of the proposed approach have been substantiated via the use of case studies, simulations, and real-world applications.

## 6 Effect of parametric uncertainty

Parametric uncertainty pertains to the intrinsic variability or limited precision of information on certain essential parameters inside a given system. In the realm of Microgrid optimization, the presence of parametric uncertainty may have notable ramifications for the design and efficacy of energy storage systems. This section provides a comprehensive analysis of the influence of parametric uncertainty on Microgrid operation.

*Performance Variability***:** The presence of parametric uncertainty may lead to fluctuations in the performance of renewable energy sources, such as changes in wind speed or solar irradiation. The aforementioned uncertainties have a direct impact on the capacity for power production and the intermittent nature of various energy sources. Therefore, it is important to take into account the many potential values of these unknown characteristics when determining the most suitable dimensions and functioning of energy storage devices. Refraining from considering this unpredictability might result in efficient storage arrangements and improved overall performance.

The occurrence of an energy imbalance in Microgrids might be attributed to parametric errors associated with load demand estimates or renewable energy output. For example, variations in load demand or unforeseen fluctuations in the supply of renewable energy might lead to an excess or shortage of energy. Energy storage systems are of utmost importance in addressing the disparity between energy supply and demand. They effectively mitigate this issue by storing surplus energy during times of low demand and then supplying more energy during periods of high demand or low energy output. Nevertheless, if the energy storage system fails to account for uncertainties sufficiently, In that case, it may need to be improved for efficiently managing energy imbalances, resulting in heightened dependence on non-renewable backup sources or possible energy inefficiencies.

The economic viability of Microgrids is contingent upon a precise assessment of operational expenses and sources of income. The financial performance of Microgrids may be greatly affected by parametric uncertainties related to variables such as power pricing, fuel costs, and government subsidies. For instance, if the prevailing power rates surpass initial projections or if there are unanticipated changes in government regulations, the economic feasibility of the Microgrid might potentially be undermined. The inclusion of these variables in the energy storage optimization process is of utmost importance in order to guarantee both resilience and financial viability.

*System Resilience*: Microgrids are often designed with the capability to function independently and endure disruptions or malfunctions inside the main grid. The presence of parametric uncertainty may have an impact on the system's capacity to effectively react to and recover from these occurrences. In the event of an unforeseen surge in load demand or a reduction in renewable energy output caused by unanticipated factors, it is important for the energy storage system to possess the potential to offset the deficit and uphold the stability of the Microgrid. Refraining from considering these uncertainties in designing and implementing energy storage systems might result in diminished system resilience and the possibility of power supply interruptions.

Parametric uncertainties possess significance for strategic planning and investment choices about the extension or enhancement of Microgrids in the long future. The ideal scale, location, and kind of energy storage systems to be installed might be influenced by uncertainties in characteristics, such as load growth rates, available land area, or future technical improvements. The use of robust optimization approaches that account for various situations and probability distributions of unknown parameters might facilitate the formulation of well-informed choices aimed at maximizing the flexibility and adaptability of the Microgrid.

In order to tackle the difficulties presented by parametric uncertainty, scholars have put forward a range of methodologies. Stochastic optimization approaches, such as robust optimization, scenario-based optimization, and chance-constrained optimization are capable of effectively managing uncertainties and delivering robust solutions in a systematic manner. These methodologies provide for examining several potential situations and implementing probabilistic modeling to account for unknown factors. The use of sensitivity analysis is also applicable in the identification of essential parameters and the assessment of their influence on the operation of a system across varying degrees of uncertainty.

In summary, the presence of parametric uncertainty presents notable obstacles to the optimization of Microgrids, particularly with regard to energy storage. It is crucial to include a comprehensive analysis of uncertainties pertaining to renewable energy output, load demand, economic variables, and system resilience in order to develop energy storage designs that are both resilient and efficient. By using stochastic optimization methods and performing sensitivity assessments, Microgrid planners and operators may enhance their decision-making process, improving the dependability, cost efficiency, and long-term sustainability of Microgrid systems.

The inclusion of uncertainty in the evaluation of energy storage performance enhances the comprehensiveness and realism of comparison techniques used in Microgrid systems. In the absence of uncertainty, deterministic optimization strategies may fail to accurately capture the inherent variety and unpredictability present in real-world scenarios. Stochastic optimization approaches, such as Monte Carlo simulation or scenario-based optimization, provide valuable insights into the efficiency of energy storage systems in the presence of varying degrees of uncertainty. The evaluation of uncertainty is contingent upon the assessment of performance measures, including robustness, risk management, and value of information. Sensitivity analysis is a valuable tool for identifying and assessing significant uncertainties within a given model, hence providing guidance for the selection and implementation of appropriate modeling methodologies. The efficacy of comparison techniques is contingent upon the unique environment in which they are used. Therefore, it is advisable to do case-specific investigations and validation procedures using real-world data.

## 7 Discussion

This paper investigates the Amended Multi-Verse Optimizer Algorithm (AMVOA) for maximizing energy storage in Microgrids. The goal is to design Microgrids with energy storage that minimizes overall cost while ensuring reliability and sustainability. The study evaluates two scenarios: Wind, PV, DG, and BESS and PV, DG, and BESS, comparing the results with other optimization algorithms.

In Scenario 1, the AMVOA algorithm successfully incorporates 84.86 % renewable energy sources while maintaining high electricity availability and meeting limitations like LPSP (5.22 %). The convergence curve and power output curves demonstrate the efficiency and effectiveness of the AMVOA algorithm in managing power generation and customer satisfaction.

In Scenario 2, the AMVOA algorithm shows promising performance in designing Microgrids with energy storage, outperforming other optimization algorithms in terms of convergence speed and solution quality. However, further analysis and consideration of specific requirements, constraints, and objectives of the HRES system are necessary to evaluate the robustness and practicality of the sizing solutions obtained by the AMVOA algorithm in real-world applications.

The investigation conducted on the optimization of energy storage solutions in Microgrids via the utilization of the AMVOA algorithm has produced encouraging outcomes and offers significant contributions to the field. This part aims to provide an explanation of the causes for the acquired results, emphasize the importance of the findings, and give a thorough and rigorous examination of the study outputs.

Several major discoveries were made while comparing two scenarios: one scenario that included wind, photovoltaic (PV), diesel, and battery power, and another scenario that exclusively used PV, diesel, and battery power. The integration of wind as a sustainable energy resource inside the Microgrid resulted in an elevated level of energy production, thereby enhancing the capacity for energy storage. This discovery is consistent with other studies that suggest wind power has the potential to make a substantial contribution to the entire energy portfolio, particularly in regions characterized by advantageous wind conditions.

Additionally, the efficacy of the AMVOA algorithm in optimizing energy storage for the purpose of attaining a harmonious equilibrium between cost optimization and reliability preservation in Microgrids was proven. The AMVOA algorithm offered novel solutions that decreased the cost of the system while achieving performance criteria via the consideration of load demand, energy storage technologies, and renewable energy sources. The program demonstrated a capacity to replicate natural phenomena and investigate various solutions within the theoretical framework of the Multi-Verse theory; therefore, presenting an innovative methodology for Microgrid design.

Additionally, the investigation underscored the need for effective energy storage management inside Microgrids. Energy storage devices have played a vital role in addressing the issue of intermittency associated with renewable energy sources and maintaining a consistent and dependable power supply during times characterized by high demand or low output. The optimization of energy storage systems' capacity and operation has led to many benefits, including better stability, less dependence on non-renewable sources, and improved cost-effectiveness.

The study also underscored the need to take into account many elements during the design process of Microgrid setups. The optimization of energy storage use may be enhanced by the integration of demand response mechanisms and load control algorithms, which effectively modify energy consumption patterns. This strategy has the potential to mitigate peak demand, alleviate strain on the Microgrid, and enhance the overall performance of the system.

The study provided a thorough examination of the optimum Microgrid designs; nonetheless, there are some aspects that require more exploration. Future research should investigate the potential integration of supplementary renewable energy sources, such as biomass, hydropower, or tidal energy in order to attain heightened degrees of sustainability. The assessment of various energy storage technologies, such as pumped hydro storage and compressed air energy storage, presents potential alternative options that possess distinct benefits in terms of scalability, efficiency, and environmental effect.

Future studies should also take into consideration the practical limitations and uncertainties that exist in real-world scenarios. The use of probabilistic modeling and stochastic optimization methods may facilitate the creation of resilient Microgrid systems that can effectively adapt to fluctuations in weather conditions, energy consumption, and fuel costs. Furthermore, it is vital to take into account economic analyses and policy consequences in order to bolster decision-making procedures pertaining to investment, pricing systems, and regulatory frameworks.

It is important to recognize and accept the inherent limits of the research study. The research was conducted with particular assumptions and limits, and the results may alter dependent on the unique attributes of various Microgrid systems. Field testing and validation are crucial procedures that serve to verify the feasibility and efficacy of the suggested designs when used in real-world scenarios.

In summary, the study results underscore the potential of the AMVOA algorithm in enhancing the efficiency of energy storage in Microgrids. The integration of wind power and efficient energy storage management has favorable prospects for attaining sustainable, dependable, and economically viable Microgrid operations. The current discourse offers a complete analysis that serves as a basis for future scholarly inquiries. It gives valuable insights into the amalgamation of diverse renewable sources, demand response tactics, different storage technologies, uncertainties, and the policy ramifications associated with these aspects. By considering and examining these many factors, we may facilitate the extensive implementation of Microgrids and make a significant contribution toward achieving a sustainable and robust energy landscape.

## 8 Conclusion

Microgrids have become a feasible option for tackling the complexities of power networks, namely in the realm of Combined Cooling Heating and Power (CCHP) systems. Localized energy systems provide a means for decentralized power production and delivery, integrating renewable energy sources and energy storage technologies to improve stability and efficiency. Energy storage is an essential component within Microgrids as it serves to address the issue of intermittency associated with renewable energy sources. By effectively storing energy, it enables the provision of a consistent power supply during times characterized by either high demand or low output. The optimization of Microgrid operations, in terms of cost and sustainability, relies heavily on the efficient management of energy storage. In order to optimize energy storage management in Microgrids, scholars have investigated the use of metaheuristic optimization methods. These algorithms provide novel solutions by emulating natural processes and identifying optimum configurations that reduce the cost of the system while satisfying performance criteria. The present study proposed a new mythology based on a modified metaheuristic called the Amended Multi-Verse Optimizer Algorithm (AMVOA), which draws inspiration from the multiverse idea. The proposed AMVOA algorithm integrated concepts from multiverse theory with metaheuristic optimization methodologies in order to provide novel approaches for the design of Microgrids. The objective of the research conducted in this study was to optimize energy storage in Microgrids via the use of the AMVOA algorithm. The research examines and contrasts two scenarios: one that integrates wind, Photovoltaic (PV), diesel, and battery power, and another that only relies on PV, diesel, and battery power. The study endeavors to provide insights into the feasibility, efficacy, and cost-efficiency of Microgrid designs with optimal energy storage systems. It will be achieved by a comprehensive analysis that encompasses cost optimization, reliability assessment, and performance evaluation. To validate the superiority of the proposed method, the method was compared with five algorithms, including the Evolutionary Algorithm (EA), Modified Grasshopper Optimization Algorithm (MGOA), Improved Gray Wolf Optimization Algorithm (IGWOA), Improved Arithmetic Optimization Algorithm (IAOA), and the original MVOA. The study compared two scenarios: one with wind, PV, diesel, and battery power and the other with only PV, diesel, and battery power. In scenario 1 (Wind, PV, DG, and BESS), optimal results were obtained using the AMVOA algorithm, resulting in a Net Present Cost (NPC) of $299,010 and an energy cost of $0.2309 per kilowatt-hour. The proposed technique successfully incorporated a significant amount of renewable energy sources (84.86 %) into the system while meeting defined limitations, such as a 5.22 % Loss of Power Supply Probability (LPSP). The optimal sizing suggested a Photovoltaic area of 155.8 $m^{2}$, a swept wind area of 263.4 $m^{2}$, a Battery Energy Storage System (BESS) capacity of 12.89 kWh, and a nominal diesel power of 17.89 kW. In scenario 2 (PV, DG, and BESS), the AMVOA algorithm provided an optimum project investment plan with a cost of $333,800 and an energy cost of $0.3451 per kilowatt-hour. The optimal sizing indicated a Photovoltaic area of 243.8 $m^{2}$ and a required diesel capacity of 18.19 kW. In this case, a Battery Energy Storage System (BESS) was not required, but the trade-offs between cost and system stability needed to be considered. The research concluded that the AMVOA algorithm outperformed other algorithms in terms of convergence and provided efficient power management in both scenarios. However, further analysis and evaluation were necessary to assess the robustness, practicality, and reliability of the proposed Microgrid configurations. The findings demonstrated the superiority of the suggested strategy when results were contrasted with those obtained using alternative optimization approaches. Future research should explore integrating renewable energy sources, demand response strategies, and evaluating different storage technologies. Real-world constraints and uncertainties should be considered, and economic analysis and policy implications should be considered. Field testing and validation of optimized energy storage solutions will validate the effectiveness and practicality of proposed designs. It will contribute to sustainable, reliable, and cost-effective Microgrid systems supporting clean and resilient energy of future.

## Data availability statement

No data was used for the research described in the article.

## CRediT authorship contribution statement

**Qingpu Hu:** Formal analysis, Software, Writing – review & editing. **Guoxin Zhao:** Conceptualization, Funding acquisition, Resources, Software. **Jian Hu:** Conceptualization, Data curation, Formal analysis, Methodology, Resources, Software. **Navid Razmjooy:** Conceptualization, Data curation, Formal analysis, Resources, Writing – original draft, Writing – review & editing.

## Declaration of competing interest

The authors declare that they have no known competing financial interests or personal relationships that could have appeared to influence the work reported in this paper.
